The article "Targeting a novel LncRNA SNHG15/miR-451/c-Myc signaling cascade is effective to hamper the pathogenesis of breast cancer (BC) in vitro and in vivo" was retracted in 2023. Reasons: duplicated images; overlap with earlier publications; signs of a paper mill; unreliable results or conclusions.

# Targeting a novel LncRNA SNHG15/miR-451/c-Myc signaling cascade is effective to hamper the pathogenesis of breast cancer (BC) in vitro and in vivo

**DOI:** 10.1186/s12935-021-01885-0

**Published:** 2021-03-31

**Authors:** Jiang Du, Hong Zhong, Binlin Ma

**Affiliations:** Department of Breast and Thyroid Surgery, The 3rd Affiliated Teaching Hospital of Xinjiang Medical University (Affiliated Cancer Hospital), Suzhou East Street No. 789, Xinshi District, Urumqi, 830011 Xinjiang China

**Keywords:** LncRNA SNHG15, Breast cancer, C-Myc, MiR-451, Malignant phenotypes

## Abstract

**Background:**

To our knowledge, LncRNA SNHG15 exerted its tumor-promoting effects to facilitate the development of breast cancer (BC), but there still needed more data to elucidate the potential underlying mechanisms.

**Methods:**

We examined genes expression status by performing Real-Time qPCR and Western Blot analysis, and cellular functions, including cell proliferation, viability, apoptosis, mobility, were measured by using the CCK-8 assay, colony formation assay, trypan blue staining assay, flow cytometer (FCM), transwell assay and wound scratch assay, respectively. The predicted targeting sites in LncRNA SNHG15, miR-451 and c-Myc 3′UTR were validated by dual-luciferase reporter gene system assay. Finally, we established the tumor-bearing mice models, and the expression status, including its enrichment and cellular localization were examined by immunohistochemistry (IHC) assay.

**Results:**

Our data indicated LncRNA SNHG15 upregulated c-Myc to facilitate BC progression by sponging miR-451 in a competing endogenous RNA (ceRNA)-dependent manner in vitro and in vivo. Specifically, LncRNA SNHG15 and c-Myc were upregulated, while miR-451 was downregulated in BC cells and clinical tissues, compared to their normal counterparts. In addition, miR-451 negatively correlated with LncRNA SNHG15 and c-Myc, and LncRNA SNHG15 was positively relevant to c-Myc in BC tissues. Next, we validated that LncRNA SNHG15 sponged miR-451 to upregulate c-Myc in BC cells. Further gain- and loss-of-function experiments evidenced that LncRNA SNHG15 promoted, while miR-451 inhibited malignant phenotypes, including cell proliferation, viability, migration, invasion and epithelial-mesenchymal transition (EMT) in BC cells. Interestingly, the inhibiting effects of LncRNA SNHG15 ablation on BC progression were abrogated by both silencing miR-451 and overexpressing c-Myc.

**Conclusions:**

We concluded that targeting the LncRNA SNHG15/miR-451/c-Myc signaling cascade was novel to hamper BC progression, which broadened our knowledge in this field, and provided potential biomarkers for BC diagnosis and treatment.

The article "Targeting a novel LncRNA SNHG15/miR-451/c-Myc signaling cascade is effective to hamper the pathogenesis of breast cancer (BC) in vitro and in vivo" was retracted in 2023. Reasons: duplicated images; overlap with earlier publications; signs of a paper mill; unreliable results or conclusions.

**Supplementary Information:**

The online version contains supplementary material available at 10.1186/s12935-021-01885-0.

## Background

Breast cancer (BC) is a huge health burden for women worldwide [1, 2], although great advances had been reached in early diagnosis and treatment therapies, BC in some patients still developed into metastatic stage and caused high mortality and worse prognosis [3–5]. Based on the previous publications [1, 2], researchers agreed that uncovering the underlying mechanisms of BC pathogenesis and developing new BC associated biomarkers became urgent and necessary for BC treatment in clinic. Recently, researchers identified that long-non coding RNAs (LncRNAs) functioned as oncogenes and tumor suppressors to modulate BC progression [6–8], and targeting LncRNAs was effective to inhibit malignant phenotypes in BC [9, 10]. Among all the LncRNAs, LncRNA SNHG15 acted as an oncogene to promote cancer development in multiple cancer types, such as lung cancer [11], prostate cancer [12], colorectal cancer [13], BC [14], etc. Specifically, Kong et al. noticed that LncRNA SNHG15 promoted BC proliferation, migration and invasion [14]. However, the detailed mechanisms of LncRNA SNHG15 in regulating BC progression are still largely unknown, hence investigations on this issue were meaningful and necessary.

MicroRNAs (miRNAs) are a group of small non-coding RNAs with about 22 nucleotides, which involved in regulating cancer progression [15, 16]. Specifically, multiple miRNAs had been identified to regulate BC pathogenesis, such as miR-200c-3p [17], miR-203a-3p [18], miR-451 [19, 20], etc. Interestingly, by performing online starBase software (http://starbase.sysu.edu.cn/), our team noticed that there existed potential targeting sites between miR-451 and LncRNA SNHG15, and previous work also validated that LncRNA SNHG15 sponged miR-451 to exert its biological functions in lung adenocarcinoma (LUAD) in a competing endogenous RNA (ceRNA) mechanism dependent manner [21], which rendered the possibility that LncRNA SNHG15 might regulate BC progression through miR-451. In addition, miR-451 served as a tumor suppressor to hamper cancer progression in multiple cancers, such as lung cancer [22], colon cancer [23], glioma [24], etc. Although previous data had suggested that miR-451 was closely related with BC pathogenesis [19, 20], the detailed mechanisms are not fully delineated.

According to the previous literatures, miRNAs always regulated cell functions through targeting the 3′ untranslated regions (3′UTRs) of their downstream targets, resulting in the degradation of these genes [25, 26]. Given the fact that miRNAs targeted 3′UTRs of cancer associated genes, by screening the existed publications in the online Pubmed database (https://pubmed.ncbi.nlm.nih.gov/), we noticed that c-Myc was proved to be the downstream target of miR-451 [27, 28], and researchers found that miR-451 targeted c-Myc to promote the development of bladder cancer [27] and lung adenocarcinoma [28], but the role of miR-451/c-Myc axis in regulating BC progression is still unknown. In addition, c-Myc acted as a proto-oncogene in BC, and Ho Yeon Lee et al. found that c-Myc driven BC metastasis to brain [29], suggesting that c-Myc was crucial for regulating BC metastasis.

The article "Targeting a novel LncRNA SNHG15/miR-451/c-Myc signaling cascade is effective to hamper the pathogenesis of breast cancer (BC) in vitro and in vivo" was retracted in 2023. Reasons: duplicated images; overlap with earlier publications; signs of a paper mill; unreliable results or conclusions.

Based on the existed information, by conducting in vitro and in vivo experiments, this study proposed to investigate the role of LncRNA SNHG15/miR-451/c-Myc signaling cascade in regulating BC progression, and uncover the possible underlying mechanisms, which will broaden our knowledge in this filed, and provide potential diagnostic and prognostic biomarkers for BC in clinic.

## Methods

### Collection and analysis of clinical samples

The BC clinical tissues and their corresponding normal adjacent tissues (N = 30) were collected in the 3rd Affiliated Teaching Hospital of Xinjiang Medical University (Affiliated Cancer Hospital) from 2014 to 2018, and the above tissues were stored at – 70 ℃ conditions immediately. The participates did not accept any treatments before surgical resection. All the clinical experiments were approved by the Ethics Committee of the 3rd Affiliated Teaching Hospital of Xinjiang Medical University (Affiliated Cancer Hospital), and the informed consent had been obtained from all the participants.

### Cell culture and vectors transfection

The BC cell lines (MDA-MB-231, MCF7, SK-BR3 and T-47D) and normal human breast epithelial cell line MCF10A were purchased from American Type Culture Collection (ATCC). The above cells were maintained in the Dulbecco’s Modified Eagle’s medium (DMEM, Gibco, USA) containing 10% fetal bovine serum (FBS, Gibco, USA), and the cells were cultivated in an incubator with humidified atmosphere containing 5% CO_2_ at 37 ℃. The overexpression and downregulation vectors for LncRNA SNHG15, miR-451 mimic and inhibitor, and c-Myc overexpression vectors were designed and synthesized by Sangon Biotech (Shanghai, China) according to the previous publications [11, 22, 28], and the Lipofectamine™ 2000 transfection reagent (Invitrogen, USA) in keeping with the manufacturer’s protocol.

### Real-Time qPCR

The total RNA was extracted from BC tissues and cells by using the commercial TRIzol reagent (Invitrogen, USA) according to the producer’s protocol. Next, LncRNA SNHG15, miR-451 and c-Myc mRNA were reversely transcribed by using the SuperScript III First-Strand Synthesis System for RT-PCR (Invitrogen, USA) and TaqMan MicroRNA Reverse Transcription Kit (Applied Biosystems, USA), respectively. Finally, the relative expression levels of the associated genes were determined by using the commercial SYBR Green PCR MasterMix (Applied Biosystems, USA) based on the instructions provided by the producer. LncRNA SNHG15 and c-Myc were normalized by β-actin, and miR-451 was normalized by U6. The primer sequences were designed according to the previous publications [11, 22, 28].

The article "Targeting a novel LncRNA SNHG15/miR-451/c-Myc signaling cascade is effective to hamper the pathogenesis of breast cancer (BC) in vitro and in vivo" was retracted in 2023. Reasons: duplicated images; overlap with earlier publications; signs of a paper mill; unreliable results or conclusions.

### Western blot analysis

The RIPA lysis buffer (Beyotime, Shanghai, China) was purchased to extract and purify the total protein from BC cells and tissues, and Western Blot analysis was conducted to examine the expression levels of c-Myc and N-cadherin based on the experimental procedures provided by the previous studies [6–8], which were normalized by β-actin. The primary antibodies against c-Myc (1:1500, Abcam, UK), N-cadherin (1:1500, Abcam, UK), Vimentin (1:2000, Abcam, UK) and β-actin (1:2000, Abcam, UK).

### Dual-luciferase reporter gene system

According to the experimental procedures provided by the previous publications [6–8], we used the online starBase software (http://starbase.sysu.edu.cn/) to predict the targeting sites among LncRNA SNHG15, miR-451 and 3′ UTRs of c-Myc mRNA, which were validated by the following dual-luciferase reporter gene system assay. Briefly, the targeting sites in LncRNA SNHG15 and c-Myc mRNA were mutated and were named as Mut-SNHG15 and Mut-Myc, respectively, and the corresponding wild-type genes were named as Wt-SNHG15 and Wt-Myc. Next, the above sequences were cloned into the pmirGLO Expression vectors (Sangon Biotech, Shanghai, China), and co-transfecting with miR-451 mimic and inhibitor into the BC cells by using the Lipofectamine™ 2000 transfection reagent. Finally, the dual-luciferase reporter gene system (Promega, USA) was employed to examine the relative luciferase activities.

### Cell counting kit-8 (CCK-8) assay

The BC cells were subjected to differential vectors transfection, and cell proliferation was measured by using the commercial CCK-8 kit purchased from YEASEN (Shanghai, China) based on the experimental procedures provided by the producer. Briefly, the cells were cultured in the 96-well plates under standard culturing conditions for 0 h, 24 h, 72 h and 96 h, and were incubated with CCK-8 reaction reagent for 2 h in the incubator. After that, the plates were shattered and the optical density (OD) values were measured at the wavelength of 450 nm to reflect relative cell proliferation abilities.

### Colony formation assay

The BC cells were pre-transfected with different vectors, and were seeded into the 24-well plates at the density of 1000 cells per well. Next, the cells were cultured in the incubator with standard culturing conditions for 14 days to form colonies. After that, the plates were stained with crystal violet (Beyotime Technology, Shanghai, China) for 15 min at room temperature. The light microscope was used to observe and photograph the colonies, and the colonies containing at least 10 cells were counted to reflect BC cell growth.

The article "Targeting a novel LncRNA SNHG15/miR-451/c-Myc signaling cascade is effective to hamper the pathogenesis of breast cancer (BC) in vitro and in vivo" was retracted in 2023. Reasons: duplicated images; overlap with earlier publications; signs of a paper mill; unreliable results or conclusions.

### Annexin V-FITC/PI double staining assay

The commercial apoptosis detection kit (HaiGene Corporation, China) was purchased to examine cell apoptosis in keeping with the manufacturer’s protocol. Briefly, the BC cells were sequentially stained with Annexin V-FITC and PI for 25 min at room temperature without light exposure. After that, a flow cytometer (ThermoFisher Scientific, USA) was employed to measure cell apoptosis ratio.

### Transwell assay

The vectors were delivered into BC cells, and the transwell assay was performed to determine cell invasion abilities. Briefly, the BC cells were cultured in the upper chamber of transwell plates (Corning Co-Star, USA) in the serum-free DMEM medium (Gibco, USA), at the density of 2 × 10^4^ cells/well. The lower chamber in the transwell system was added with DMEM medium containing 10% fetal bovine serum (FBS, Gibco, USA). At 24 h post-culture, the filters were fixed by using the 4% paraformaldehyde and stained by 0.1% crystal violet for visualization. Finally, the cells were photographed by the light microscope, and cell number was counted to reflect cell invasion abilities.

### Wound scratch assay

The BC cells were cultivated in the 6-well plates at the density of 6 × 10^5^ cells per plate, and the cells were cultured under standard conditions until the cell confluency reached 100%. After that, the 200 pipette tips were used to equally generate the wound scratches, and the plates were placed back to the incubator and the cells were observed every day by using the light microscope. The scratch distance was calculated to reflect relative cell migration abilities.

### Establishment of xenograft tumor-bearing mice models

The nude mice (6–8 weeks) were purchased from the animal center of the Xinjiang Medical University and were fed under the standard conditions. The BC cells were subcutaneously injected into the back flank of nude mice at the concentration of 5 × 10^6^ cells per mouse, each group had 5 mice, and the mice were fed under the standard conditions. At 25 days post-injection, the mice were anesthetized by intravenously injecting Barbiturate at the concentration of 100 mg/kg, and the standards for successful euthanasia included: (1) no cardiac arrest; (2) no spontaneous breath for at least 3 min; and (3) no blinking reflex in mice. Subsequently, the mice were sacrificed, the mice tumors were isolated and weighed to reflect tumorigenesis. Each group included at least 3 mice. All the animal experiments were approved by the Ethics Committee of the 3rd Affiliated Teaching Hospital of Xinjiang Medical University (Affiliated Cancer Hospital).

The article "Targeting a novel LncRNA SNHG15/miR-451/c-Myc signaling cascade is effective to hamper the pathogenesis of breast cancer (BC) in vitro and in vivo" was retracted in 2023. Reasons: duplicated images; overlap with earlier publications; signs of a paper mill; unreliable results or conclusions.

### Immunohistochemistry (IHC)

The mice tumor tissues were prepared and sliced into sections, the IHC was conducted to determine the expression patterns (expression levels and localization) of Ki67 protein in the tissues. The Ki67 protein antibody was purchased from Abcam (1:400, #ab245113, UK), and the detailed experimental procedures for IHC were well recorded in the previous publications [6–8].

### Data collection and analysis

The data was presented as Means ± Standard Deviation (SD), and SPSS 18.0 software was used to analyze the statistical significance. Specifically, the Student’s t-test was used for the comparisons between two groups, and the one-way ANOVA analysis was conducted to compare the means from multiple groups. In addition, the Pearson correlation analysis was used to analyze the correlations of genes expressions in the clinical samples. *P < 0.05 was regarded as statistical significance. Each experiment was triplicated.

## Results

### Upregulated LncRNA SNHG15 and c-Myc, and downregulated miR-451 were observed in BC cells and tissues

The cancerous and their paired normal adjacent tissues were collected from BC patients (N = 30), and the expression status of LncRNA SNHG15, miR-451 and c-Myc were determined by Real-Time qPCR and Western Blot. As shown in Fig. 1a–c, the data indicated that the expression levels of LncRNA SNHG15 (Fig. 1a) and c-Myc mRNA (Fig. 1c) were increased, while miR-451 (Fig. 1b) was decreased in cancer tissues, instead of their paired normal tissues. Consistently, the 4 paired clinical samples were randomly selected from the patients, and the results validated that c-Myc was also upregulated in BC tissues at translated levels (Fig. 1d). Also, data from TCGA database suggested that the breast invasive carcinoma (BRCA) patients with high-LncRNA SNHG15 tended to have a worse prognosis (Additional file 1: Figure S1). Next, by conducting the Pearson correlation analysis, we evidenced that miR-451 was negatively related to both LncRNA SNHG15 (Fig. 1e) and c-Myc mRNA (Fig. 1f), while the expression levels of LncRNA SNHG15 and c-Myc mRNA showed positive correlations in BC tissues (Fig. 1g). Furthermore, the BC cell lines (MDA-MB-231, MCF7, SK-BR3 and T-47D) and normal human breast epithelial cell line MCF10A were obtained and analyzed (Fig. 1h–k). As expected, LncRNA SNHG15 (Fig. 1h) and c-Myc (Fig. 1j, k) were prone to be high-expressed, but miR-451 tended to be low-expressed in BC cells (Fig. 1i), in contrast with the normal MCF10A cells. Since LncRNA SNHG15 was especially upregulated in MDA-MB-231 and MCF7 cells, instead of the SK-BR3 and T-47D cells (Fig. 1h), we selected the two cell lines for further investigations.

The article "Targeting a novel LncRNA SNHG15/miR-451/c-Myc signaling cascade is effective to hamper the pathogenesis of breast cancer (BC) in vitro and in vivo" was retracted in 2023. Reasons: duplicated images; overlap with earlier publications; signs of a paper mill; unreliable results or conclusions.

**Fig. 1:** LncRNA SNHG15, miR-451 and c-Myc were aberrantly expressed in BC clinical specimens and cells. The BC tissues and their paired adjacent normal tissues were collected, and Real-Time qPCR was conducted to determine the expression levels of (**a**) LncRNA SNHG15, (**b**) miR-451 and (**c**) c-Myc mRNA. **d** Western Blot analysis was employed to examine c-Myc protein levels in the clinical tissues. **e**–**g** Pearson correlation analysis was used to analyze the correlations among LncRNA SNHG15, miR-451 and c-Myc in BC tissues. The BC cell lines (MDA-MB-231, MCF7, SK-BR3 and T-47D) and normal human breast epithelial cell line MCF10A were cultured in vitro, and the expression levels of (**h**) LncRNA SNHG15, (**i**) miR-451 and (**j**) c-Myc mRNA were determined by Real-Time qPCR. **k** The c-Myc protein expressions in the cells were measured by using the Western Blot analysis. Each experiment repeated at least 3 times, and *P < 0.05 indicated statistical significance

### LncRNA SNHG15 sponged miR-451 to upregulate c-Myc in BC cells

Based on the information from the online starBase software (http://starbase.sysu.edu.cn/) and the data from the previous publications [27, 28], we assured that miR-451 potentially bound to LncRNA SNHG15 (Fig. 2a) and 3′ untranslated region (3′UTR) of c-Myc mRNA (Fig. 2d). Next, the wild-type targeting sites in LncRNA SNHG15 (Wt-SNHG15) and 3′ UTR of c-Myc (Wt-Myc) were mutated, and they were named as Mut-SNHG15 and Mut-Myc, respectively, the dual-luciferase reporter gene system assay results indicated that the relative luciferase activity was decreased by miR-451 mimic, and was increased by miR-451 inhibitor in BC cells co-transfecting with Wt-SNHG15 (Fig. 2b, c) and Wt-Myc (Fig. 2e, f), instead of their corresponding mutant counterparts, suggesting that we had validated the binding sites among LncRNA SNHG15, miR-451 and c-Myc. Furthermore, the overexpression and downregulation vectors for LncRNA SNHG15 (Additional file 3: Figure S3A) and miR-451 (Additional file 3: Figure S3B) were delivered into BC cells, and we evidenced that LncRNA SNHG15 positively regulated (Fig. 2g–i), while miR-451 negatively modulated c-Myc in BC cells (Fig. 2j–l). Also, further data suggested that the inhibiting effects of LncRNA SNHG15 ablation on c-Myc expressions were reversed by downregulating miR-451 (Fig. 2m–o), suggesting that knockdown of LncRNA SNHG15 suppressed c-Myc through releasing miR-451 in BC cells.

The article "Targeting a novel LncRNA SNHG15/miR-451/c-Myc signaling cascade is effective to hamper the pathogenesis of breast cancer (BC) in vitro and in vivo" was retracted in 2023. Reasons: duplicated images; overlap with earlier publications; signs of a paper mill; unreliable results or conclusions.

**Fig. 2:** The regulatory mechanisms of LncRNA SNHG15, miR-451 and c-Myc were investigated. The online starBase software (http://starbase.sysu.edu.cn/) was employed to predict the binding sites of miR-451 with (**a**) LncRNA SNHG15 and (**d**) 3′UTR of c-Myc mRNA. Dual luciferase reporter gene system was performed to validate the targeting sites of miR-451 with (**b**, **c**) LncRNA SNHG15 and (E, F) 3′UTR of c-Myc mRNA in BC cells. By performing Real-Time qPCR and Western Blot, we evidenced that (**g–i**) LncRNA SNHG15 positively regulated c-Myc, and (**j–l**) miR-451 negatively regulated c-Myc in BC cells. In addition, (**m**–**o**) silencing of LncRNA SNHG15 inhibited c-Myc expressions through releasing miR-451. Each experiment repeated at least 3 times, and *P < 0.05 indicated statistical significance

### The role of LncRNA SNHG15 in regulating malignant phenotypes in BC cells

Previous data suggested that LncRNA SNHG15 functioned as an oncogene to accelerate BC progression [14], which were validated by our work. As shown in Fig. 3a, b, upregulation of LncRNA SNHG15 promoted cell proliferation in BC cells, which were inhibited by downregulating LncRNA SNHG15. Consistently, the colony formation assay results validated that LncRNA SNHG15 also positively regulated colony formation abilities in BC cells (Fig. 3c, d). Next, the Annexin V-FITC/PI double staining assay was used to examine cell apoptosis, and the results in Fig. 3e, f showed that knock-down of LncRNA SNHG15 triggered apoptotic cell death in BC cells. In addition, we noticed that upregulated LncRNA SNHG15 increased the expression levels of N-cadherin (Fig. 3g) and Vimentin (Additional file 2: Figure S2A–D), but inhibited E-cadherin (Additional file 2: Figure S2A–D) to promote epithelial-mesenchymal transition (EMT), and silencing of LncRNA SNHG15 had opposite effects (Fig. 3g, Additional file 2: Figure S2A–D). Furthermore, LncRNA SNHG15 overexpression promoted cell invasion (Fig. 3h) and migration (Fig. 3i) in BC cells, while LncRNA SNHG15 ablation had opposite effects on cell mobility (Fig. 3h, i).

**Fig. 3:** LncRNA SNHG15 promoted malignant phenotypes in BC cells. **a**, **b** CCK-8 assay was performed to determine cell proliferation abilities. **c, d** Colony formation assay was used to examine colonies formation abilities in BC cells. **e, f** Knock-down of LncRNA SNHG15 promoted cell apoptosis in BC cells, which were determined by using Annexin V-FITC/PI double staining method. **g** The expression levels of N-cadherin were monitored by using the Western Blot analysis. **h **Cell invasion and (**i**) migration were detected by transwell assay and wound scratch assay, respectively. Each experiment repeated at least 3 times, and *P < 0.05 indicated statistical significance

The article "Targeting a novel LncRNA SNHG15/miR-451/c-Myc signaling cascade is effective to hamper the pathogenesis of breast cancer (BC) in vitro and in vivo" was retracted in 2023. Reasons: duplicated images; overlap with earlier publications; signs of a paper mill; unreliable results or conclusions.

### MiR-451 acted as a tumor suppressor to impede BC progression

Next, we performed further experiments to investigate the role of miR-451 in regulating BC progression. To achieve this, the miR-451 mimic and inhibitor were transfected into BC cells to overexpress and downregulate miR-451 (Additional file 3: Figure S3B), and CCK-8 assay was performed to examine cell proliferation (Fig. 4a, b). As shown in Fig. 4a, b, the results showed that miR-451 negatively regulated cell proliferation in BC cells. Also, by performing the colony formation assay, we also verified that overexpression of miR-451 inhibited colony formation abilities in BC cells, but miR-451 ablation had opposite effects (Fig. 4c, d). Similarly, the data in Fig. 4e, f indicated that upregulation of miR-451 also induced cell apoptosis in BC cells. Furthermore, we proved that upregulated miR-451 inhibited N-cadherin to reverse EMT in BC cells, which could be promoted by downregulating miR-451 (Fig. 4g). Finally, our data evidenced that miR-451 overexpression inhibited cell invasion (Fig. 4h) and migration (Fig. 4i) in BC cells, while knock-down of miR-451 promoted cell mobility (Fig. 4h, i).

**Fig. 4:** MiR-451 acted as a tumor suppressor to hinder BC progression in vitro. **a**, **b** The CCK-8 assay results indicated that miR-451 inhibited BC cell proliferation. **c**, **d** The colonies formation abilities were inhibited by overexpressing miR-451 in BC cells. **e, f** The Annexin V-FITC/PI double staining assay evidenced that upregulation of miR-451 induced cell apoptosis in BC cells. **g** By performing Western Blot, we noticed that miR-451 negatively regulated N-cadherin to inhibit EMT in BC cells. Cell mobility was evaluated by using (**h**) transwell and (**i**) wound scratch assay, respectively. Each experiment repeated at least 3 times, and *P < 0.05 indicated statistical significance

### Silencing of LncRNA SNHG15 inhibited BC development by targeting miR-451 and c-Myc

Given the fact that there existed regulatory mechanisms among LncRNA SNHG15, miR-451 and c-Myc, we speculated that LncRNA SNHG15 might regulate malignant phenotypes in BC cells by targeting the miR-451/c-Myc axis. To validate this hypothesis, the LncRNA SNHG15 downregulation vectors (Additional file 3: Figure S3A), miR-451 inhibitor (Additional file 3: Figure S3B) and c-Myc overexpression vectors (Additional file 3: Figure S3C, D) were successfully transfected into BC cells, which were divided into 4 groups, including control, LncRNA SNHG15 knock-down (KD-SNHG15), KD-SNHG15 + KD-miR-451 and KD-SNHG15 + OE-Myc. The above cells were cultured under the standard conditions for 0 h, 24 h, 48 h and 72 h, respectively. The CCK-8 assay results showed that the inhibiting effects of silencing LncRNA SNHG15 on BC cell proliferation were reversed by both downregulating miR-451 and upregulating c-Myc (Fig. 5a, b), and the above results were validated by the following colony formation assay (Fig. 5c, d). Consistently, further data suggested that knock-down of LncRNA SNHG15 triggered apoptotic cell death in BC cells by regulating the miR-451/c-Myc axis in a similar manner (Fig. 5e, f). Next, the Western Blot analysis results evidenced that miR-451 ablation and c-Myc overexpression also reversed the inhibiting effects of LncRNA SNHG15 silence on N-cadherin expressions in BC cells (Fig. 5g). Finally, the BC cells were used to establish xenograft tumor bearing mice models, and the results showed that knock-down of LncRNA SNHG15 inhibited tumor growth (Fig. 6a, b) and Ki67 expressions (Fig. 6c) in mice tumor tissues to hinder tumorigenesis of BC cells in vivo, which were all reversed by both silencing miR-451 and upregulating c-Myc (Fig. 6a, c).

The article "Targeting a novel LncRNA SNHG15/miR-451/c-Myc signaling cascade is effective to hamper the pathogenesis of breast cancer (BC) in vitro and in vivo" was retracted in 2023. Reasons: duplicated images; overlap with earlier publications; signs of a paper mill; unreliable results or conclusions.

**Fig. 5:** Knock-down of LncRNA SNHG15 inhibited BC progression in vitro and in vivo by targeting miR-451 and c-Myc. **a, b** Cell proliferation was evaluated by using the CCK-8 assay. **c**, **d** Colony formation abilities were measured by conducting the colony formation assay. **e**, **f** Annexin V-FITC/PI double staining assay results suggested that silencing of LncRNA SNHG15 promoted cell apoptosis in BC cells by targeting miR-451 and c-Myc. **g** Western Blot analysis was used to detect N-cadherin expressions to determine EMT in BC cells. Each experiment repeated at least 3 times, and *P < 0.05 indicated statistical significance

**Fig. 6:** The BC cells were utilized to establish xenograft tumor-bearing mice models, and (**a**, **b**) tumor weight was measured at day 25 post-injection. **c** The immunohistochemistry (IHC) was used to examine the expressions and localization of Ki67 protein in mice tumor tissues, and the cells stained with yellow were regarded as Ki67-positive cells, which were indicated by the red arrows, and the intensity of the arrows represented relative Ki67 protein levels. Each experiment repeated at least 3 times, and *P < 0.05 indicated statistical significance

## Discussion

Although recent data had assured that LncRNA SNHG15 acted as an oncogene to promote cancer development in multiple cancers [11–14], the detailed underlying mechanisms of LncRNA SNHG15 in regulating BC pathogenesis are still not fully delineated. To investigate this issue, the present study collected clinical tissues from 30 BC patients, and validated that LncRNA SNHG15 tended to be enriched in cancer tissues, instead of their corresponding normal adjacent tissues. Consistently, high-expressed LncRNA SNHG15 was also observed in BC cells, compared to the normal MCF10A cells, indicating that LncRNA SNHG15 was aberrantly upregulated in BC cells and tissues. Next, by performing the gain- and loss-of-function experiments, we found that knock-down of LncRNA SNHG15 inhibited cell proliferation, colonies formation, epithelia-mesenchymal transition (EMT), invasion, and migration, and induced apoptotic cell death in BC cells, while LncRNA SNHG15 had opposite effects on the above malignant phenotypes. Consistently, the in vivo experiments evidenced that silencing of LncRNA SNHG15 slowed down tumor growth and inhibited Ki67 protein levels to hinder tumorigenesis of BC cells in xenograft mice models. The above results suggested that LncRNA SNHG15 promoted BC progression, which were supported by the previous work [14].

The article "Targeting a novel LncRNA SNHG15/miR-451/c-Myc signaling cascade is effective to hamper the pathogenesis of breast cancer (BC) in vitro and in vivo" was retracted in 2023. Reasons: duplicated images; overlap with earlier publications; signs of a paper mill; unreliable results or conclusions.

Previous publications indicated that miR-451 was closely associated with BC progression and prognosis [19, 20], but the detailed mechanisms are still largely unknown. The present study investigated this issue and found that miR-451 functioned as a tumor suppressor to hinder BC development in vitro. Mechanistically, miR-451 was downregulated in both BC tissues and cells, in contrast with their counterparts. Next, the miR-451 mimic and inhibitor were transfected into BC cells to overexpress and silence miR-451, respectively. As expected, the results showed that overexpression of miR-451 inhibited BC cell growth and mobility, and promoted cell apoptosis, but miR-451 downregulation facilitated BC progression, indicating that miR-451 acted as a tumor suppressor to hamper BC development, which were supported by the data in lung cancer [22], colon cancer [23], glioma [24], etc. According to the previous work [21], we validated that LncRNA SNHG15 sponged miR-451 in BC cells in a ceRNA-dependent manner, and further experiments showed that the inhibiting effects of LncRNA SNHG15 ablation on the malignant phenotypes in BC cells were all reversed by silencing miR-451, implying that LncRNA SNHG15 promoted BC progression by sponging miR-451.

Ho Yeon Lee et al. proved that the proto-oncogene c-Myc was a crucial “driver” to promote BC metastasis to brain [29], which also played an oncogenic role in multiple cancers [30–32]. Expectedly, we noticed that c-Myc tended to be overexpressed in BC tissues and cells, instead of their normal counterparts, which indirectly reflected that high-expressed c-Myc indicated a worse outcome in BC. In addition, we validated that miR-451 targeted 3′UTR of c-Myc mRNA for degradation, and LncRNA SNHG15 positively regulated c-Myc in BC cells by targeting miR-451, implying that LncRNA SNHG15 sponged miR-451 to upregulate c-Myc in BC cells. Next, we confirmed that LncRNA SNHG15 regulated BC development by upregulating c-Myc. Specifically, the inhibiting effects of LncRNA SNHG15 ablation on the malignant phenotypes in BC cells were all reversed by overexpressing c-Myc.

The article "Targeting a novel LncRNA SNHG15/miR-451/c-Myc signaling cascade is effective to hamper the pathogenesis of breast cancer (BC) in vitro and in vivo" was retracted in 2023. Reasons: duplicated images; overlap with earlier publications; signs of a paper mill; unreliable results or conclusions.

## Conclusions

Taken together, this study validated that targeting LncRNA SNHG15 impeded BC progression in vivo and in vitro by modulating the miR-451/c-Myc pathway. The present study uncovered the possible underlying mechanisms of BC development, and provided LncRNA SNHG15, miR-451 and c-Myc as novel biomarkers for BC diagnosis and prognosis.

## Supplementary Information

**Additional file 1: Figure S1.** The correlations of LncRNA SNHG15 and BRCA patients’ prognosis were analyzed by the Pan-cancer analysis, and the original data were obtained from TCGA database.

**Additional file 2: Figure S2.** Western Blot were used to examine the expression levels of E-cadherin and Vimentin in the (A, B) MDA-MB-231 cells and (C, D) MCF7 cells. Individual experiment had 3 repetitions, and *P < 0.05.

**Additional file 3: Figure S3.** Real-Time qPCR was used to examine the expression levels of (A) LncRNA SNHG15 and (B) miR-451, and Western Blot was employed to detect c-Myc expressions in the MDA-MB-231 cells and MCF7 cells. Individual experiment had 3 repetitions, and *P < 0.05.

## Data Availability

All the data involved in this study had been included in the manuscript, and the corresponding raw data could be acquired from the corresponding author upon reasonable request.

## Abbreviations

BC: Breast cancer
CCK-8: Cell counting kit-8
IHC: Immunohistochemistry
ceRNA: Competing endogenous RNA
EMT: Epithelial-mesenchymal transition
LncRNAs: Long-non coding RNAs
miRNAs: MicroRNAs
LUAD: Lung adenocarcinoma
3′UTRs: 3′ Untranslated regions
ATCC: American Type Culture Collection
FBS: Fetal bovine serum
